The article "Clinical and Imaging Study of Repetitive Transcranial Magnetic Stimulation in the Treatment of Morphine Dependence Through mGluR5/TDP43/NR2B Pathway" was retracted in 2022. Reason: concerns about the peer review.

# Clinical and Imaging Study of Repetitive Transcranial Magnetic Stimulation in the Treatment of Morphine Dependence Through mGluR5/TDP43/NR2B Pathway

**DOI:** 10.1155/2021/6733963

**Published:** 2021-10-20

**Authors:** Xin Li, Congyan Li, Jia'nan Yu, Qing Ji, Wei Wang, Ying Peng, Xiaofeng Zhu, Jiguang Liu

**Affiliations:** ^1^School of Basic Medicine, Jiamusi University, Jiamusi 154000, Heilongjiang, China; ^2^Department of Neurology, The First Affiliated Hospital of Jiamusi University, Jiamusi 154000, Heilongjiang, China; ^3^Graduate School, Jiamusi University, Jiamusi 154000, Heilongjiang, China; ^4^Department of Neurology, Sun Yat-sen Memorial Hospital, Sun Yat-sen University, Guangzhou 510000, Guangdong, China; ^5^Mudanjiang Medical University, Mudanjiang 157000, Heilongjiang, China

## Abstract

Morphine is tolerable after long-term use. After long-term use, it will have a great impact on the human body, and the treatment effect is not good. In recent years, the continuous development of repetitive transcranial magnetic stimulation (rTMS) treatment technology has made a treatment. Drug-resistant morphine dependence has a breakthrough. In this article, to study the effect of repeated transcranial magnetic stimulation in the treatment of morphine dependence through mGluR5/TDP43/NR2B pathway, experiments were carried out on rats to compare the changes in the images of rats after different periods of morphine use and their effects on morphine withdrawal. During the period, the performance of rats provides a reference for repeated transcranial stimulation to treat morphine dependence. According to the experimental results, after stopping morphine, withdrawal from the rats, irritable acts, and patience diminished. This is a decrease of more than 50% in comparison with the one of the normal group. There was a different degree of variability in the treatment images of mGluR5/TDP43 and so on after rTMS treatment, and the changes were large. These reductions in detoxification responses in rodents suggest that rTMS serves an instrumental role in the prevention and treatment of phosphorylation related to morphine dependence.

## 1. Introduction

Drug dependence refers to the phenomenon of increased tolerance, withdrawal symptoms, and mental dependence behaviors caused by the long-term use of addictive substances. At present, the drug dependence problem caused by the abuse or active use of addictive drugs is becoming more and more serious, which has caused great harm to social security and economic development. Investigations and evaluations suggest that, among countries with a high rate of illegal drug use, marijuana is the most frequently used drug with proven dependence, cocaine is the second, and amphetamine is the third; among prescription drugs approved for sale by the government, pain relief drugs, sedatives, and stimulants have been severely abused and have become the main lethal drugs. Long-term use of drugs including morphine (Mor), cocaine, methamphetamine, and other dependent drugs can affect the neural pathways related to rewards, learning, and memory and cause long-term adaptive changes, such as changes in the transmitter system and disturbances in signal transduction pathways. As well as changes in synaptic plasticity, patients have a severe craving for drugs, withdrawal symptoms, and compulsive drug-seeking behavior. A complete and effective treatment plan is lacking in clinical practice, and most people have up to 95% chance of relapse when they are reexposed with the factors associated with the drug-using drug environment. Searching for effective therapeutic agents and medications to be used to treat withdrawal with symptoms of dependence and psychological cravings induced by relapse in dependent patients in this area has been a key focus and point of enquiry in this field.

The article "Clinical and Imaging Study of Repetitive Transcranial Magnetic Stimulation in the Treatment of Morphine Dependence Through mGluR5/TDP43/NR2B Pathway" was retracted in 2022. Reason: concerns about the peer review.

Until the establishment of an objective effective behavioral assessment system, it has been difficult for dependence assessing to make valid predictions. The assessment methods for studying drug addiction, for instance, have been improved by the introduction of new methodologies for assessment and by further research on objective behavior crises and mechanisms of addictive practices. At present, the commonly used internal and external dependence evaluation methods are mainly divided into two categories: physical dependence and psychological dependence. Among them, the physical dependence evaluation should include physical withdrawal experiments, impulsive withdrawal experiments, and substitution experiments. In specific cortical areas, even in the pyramidal phase of neurons, there will be repeated and regular stimulation, which can stimulate horizontal neurons and improve the function of local and remote neural networks. It can reconstruct peripheral cortex function and affect brain tissue metabolism, blood flow, and neurotransmitter transmission. In this paper, repeated transboundary magnetic stimulation of the mGluR5/TDP43/NR2B pathway was used to study the clinical response of morphine to drug treatment.

For repetitive transcranial stimulation, experts at home and abroad also have many studies. Rabey and Dobronevsky believed that transcranial magnetic stimulation is a noninvasive technique that can produce current-induced modulation in cortical excitability. Previous clinical trials have shown that the combination of rTMS and cognitive training (rTMS-COG) provided by the NeuroAD medical device system provides a novel, safe, and effective way to improve patients with mild to moderate AD. The experience of using rTMS-COG treatment in a clinical setting was introduced. 30 mild to moderate AD patients received rTMS-COG commercial treatment in two clinics, 5 days a week, 1 hour a day, for 6 weeks (30 Festivals). Five patients returned for a second treatment. ADAS-Cog scores were measured before and after treatment, confirming that rTMS can improve patients' cognition [1]. In 38 healthy, right-handed female participants, Remue et al. examined a single sham operation-controlled high-frequency (HF) repetitive transcranial magnetic stimulation (rTMS) session on the left (*n* = 19) and right (*n* = 19). The influence of the dorsolateral prefrontal cortex (DLPFC) on the stress response of the autonomic nervous system is measured by heart rate variability (HRV). Stress is induced instantaneously through evaluative negative feedback, which proves that although the induction program can effectively increase self-reported pain in all groups and conditions, only after real HF-rTMS on the left DLPFC, the physiological stress response will weaken [2]. The noninvasive language mapping performed by Ille et al. through repetitive navigational transcranial magnetic stimulation (rTMS) often shows a high correlation with the results of DCS language mapping in language negative brain regions, purely based on rTMS language mapping to analyze the oncology and functional results of patients, undergoing periscoliosis resection. Data from rTMS language mapping and rTMS-based diffusion tensor imaging fiber tracking (DTI-FT) are transmitted to the intraoperative neuronavigation system [3, 4]. These studies have a certain reference effect for this article, but due to the insufficient sample size of related studies, it is difficult to replicate, so the experimental results are not repeatable.

The article "Clinical and Imaging Study of Repetitive Transcranial Magnetic Stimulation in the Treatment of Morphine Dependence Through mGluR5/TDP43/NR2B Pathway" was retracted in 2022. Reason: concerns about the peer review.

The new and innovative aspect of it is to establish a Chronic Morphine Dependence Model on Rat based on the previous work on the evaluation of morphine dependence complex. The expression levels of mGluR5/TDP43/NR2B and the levels of gene transfer at each withdrawal point in the hemorrhoids of rats were abrogated and probed. Continuously change the inhibitory level of the promoter region of H3K9 cells and analyze withdrawal symptoms scores, mGluR5/TDP43/NR2B protein expression, and NR2B Correlation between mRNA expression of mGluR5/TDP43/NR2B promoter gene H3K9 histone inactivation level.

## 2. Clinical and Imaging Research Methods of Morphine Dependence

### 2.1. rTMS

rTMS was developed based on TMS, which gives repetitive and regular stimulation to specific cortical areas [5, 6]. The current high-frequency stimulation methods are widely used in the field of cognitive impairment, and there are many studies. It can improve the patient's attention, language function, orientation, executive function, and so forth [7].

Compared with low-frequency magnetic stimulation, high-frequency magnetic stimulation has a better effect on improving the symptoms of patients with mild to moderate dementia. However, more and more studies have found that the effects of high-frequency and low-frequency stimulation on brain function have not been completely reversed. Low-frequency stimulation also plays an important role in improving brain diffusion and restoring brain function, and it is safe in terms of safety [8]. This may be better than high-frequency stimulation. The earliest research found that low-frequency rTMS can improve the memory and function of patients with amnesia to varying degrees. There is no significant difference between the learning and memory ability of the rat MCI model and high-frequency stimulation [9]. The structure of the brain network is interconnected. Since the prefrontal cortex is a brain structure closely related to cognitive functions, this study intends to select the frontal cortex of the dominant hemisphere as the stimulation point [10, 11]. Through the treatment of 1 Hz low-frequency rTMS in the behavioral phase of MCI patients for 6 weeks, explore its recognition effect in patients with morphine dependence [12]. The degree of repetitive transcranial magnetic stimulation is shown in Figure 1.

The Montreal Cognitive Assessment Scale (MoCA) was developed by Canadian Nasreddine and others based on the cognitive items and scores of the clinical experience. The cut-off value is 26-minute sensitivity and specificity is 89% and 91%, which can fully evaluate cognitive function [11]. However, peer-reviewed evaluations are still thematic and are easily affected by factors such as the evaluator, the patient's condition, and whether the operation is standard. So, objective testing and analysis have been important for the correct and prompt diagnosis and estimation of MCI. Moreover, more and more of the biological indicators are being used continuously to aid in the diagnosis of MCI and AD as an aid, such as measurement of Tau protein and b amyloid (b) in cerebrospinal fluid, for instance, some structural and functional neuroimaging techniques, measuring brain tumors and hippocampal tumors, and detecting glucose metabolic rate in cognitive areas of the cerebrum [12]. However, the implementation cost is relatively high, most of which are only used for scientific research and have limited clinical applications. Therefore, EEG is simple, cheap, noninvasive, and safe. EEG signals contain rich neocortical activity information, reflecting the brain dynamics and brain dynamics of patients with morphine dependence in different cognitive states [13]. With this paper, the optimal stimulation profile of rTMS for morphine dependence will be investigated and searched to have a baseline for clinical treatment of morphine dependence and to provide better rehabilitation and timely guidance program for these patients as well as understanding the effect of rTMS treatment on morphine dependence.

The article "Clinical and Imaging Study of Repetitive Transcranial Magnetic Stimulation in the Treatment of Morphine Dependence Through mGluR5/TDP43/NR2B Pathway" was retracted in 2022. Reason: concerns about the peer review.

Using the rTMS mechanism, if the bilateral cerebral hemispheres are stimulated by different frequencies of rTMS, the restoration speed of the active inhibitory balance of the cerebral hemispheres may be accelerated. In this way, it can quickly reach a new and higher dynamic balance level. The accelerated degradation depends on the function. However, there has been no such report so far [14, 15]. Based on this, this article will research and find the best stimulation parameters for rTMS to treat morphine dependence, provide a baseline for the clinical treatment of morphine dependence, and provide patients with better rehabilitation and timely guidance programs, as well as understanding RTMS treatment for morphine dependence Impact.

### 2.2. Ways to Treat Morphine Dependence

The mechanism of morphine dependence is very complex and may be related to many factors such as neurobiology, psychology, and sociology. Studies have shown that more than half of the phenotypic variants associated with morphine use disorder and long-term use of morphine can lead to increased tolerance, deprivation, and craving, which indicates that human biological characteristics have changed [16–18]. However, from the perspective of genetic analysis, the genes that control these characteristics have not been mutated. One of the mechanisms may be to change the belief that the individual's susceptibility to diseases is controlled by genotypes, and the appearance and phenotype of diseases are controlled by genetic modifications decided. Genetics refers to changes based on gene expression levels. The unchanging DNA coding sequence is equivalent to changing the genetic material, not the genetic information in the cell [19]. The genotype has not changed, but the phenotype has changed. This plays a key role in adapting to changes in the environment. This regulation of gene expression that affects gene transfer activity does not involve changes in DNA sequence and is called EPI transcription regulation. It involves many complex pathological processes of human diseases, such as morphine use disorder [20].

The article "Clinical and Imaging Study of Repetitive Transcranial Magnetic Stimulation in the Treatment of Morphine Dependence Through mGluR5/TDP43/NR2B Pathway" was retracted in 2022. Reason: concerns about the peer review.

Although the position of morphine in the NMDA receptor has not been determined, it has been found that the effect of morphine on the central nervous system is related to the tolerance of the receptor, their phosphorylation position, and location, especially NR2B. Morphine treatment of mice with less than 25 mM can significantly inhibit NR2B, and a slightly higher concentration can inhibit NR2A, but even if the concentration reaches 100 mm, it has no inhibitory effect on NR2C and NR2D [21].

Studies have shown that the main mode of action of morphine on NMDA receptors may be NR2B, mainly an increase in NR2B mRNA levels. NR2A, NR2C, and nr2d, including NR3, are more sensitive to morphine. Preliminary experiments with animals in the experimental group also showed that the expression of NR2B in the prefrontal cortex and hippocampus of morphine-treated rats was significantly increased. During pregnancy, morphine can cause the same changes in the expression of NR2B in the relevant brain regions of the offspring of rats. Accompanying cognitive impairment and some drug interventions may help alleviate this phenomenon.

NMDA receptors play an important role in the formation of brain synapses, neuronal migration, and gene expression during embryonic development. In animals, we found that NMDA receptors overlap in part of the brain. The NR2A system is located in the central nervous system. In addition, the NR2B family is located in the central nervous system. NR2A distribution is mainly in the frontolimbic lobe, which includes the nucleus pallidus, hippocampus, and trunk cells. Substance-related brain territories mainly comprise the diaphragm, cnidium, and myelomeninges. The brain areas related to drugs mainly include the abdomen, cell nucleus, and amygdala. It is mainly concentrated not only on NR2B but also NR2B [22]. Many studies have shown that NR2A NMDA receptor subunits are mainly involved in normal opioid-induced addiction, while NR2B may be mainly involved in regulating opioid-induced mental dependence.

### 2.3. Clinical Impact

There is noise in the image that is derived from the actual surrounding environment. Characteristics of various types of noise have been made more ambiguous by various complexity and varieties of environments, both in the process of receiving and transmitting images. The quality components of the image sensing unit, the contextual conditions which surround the image acquisition, and the transmissive channel to which the image is transmitted, affect the image generation and may lead to noise in the scene [23, 24]. Mathematically speaking, according to the relationship between image and noise, noise is generally divided into two categories: multiple noise and additional noise.

The article "Clinical and Imaging Study of Repetitive Transcranial Magnetic Stimulation in the Treatment of Morphine Dependence Through mGluR5/TDP43/NR2B Pathway" was retracted in 2022. Reason: concerns about the peer review.

Impulse noise is also called salt and pepper noise. The density function of impulse noise is

(1) $$\begin{array}{c} p\left(m\right)=\left\{\begin{array}{cc} p_{a}, & m=a,\\ p_{b}, & m=b,\\ 0, & \text{other.} \end{array}\right. \end{array}$$

Gaussian noise is also called normal noise, and its probability density function is

(2) $$\begin{array}{c} p\left(m\right)=\frac{1}{\sqrt{2\pi \varepsilon }}e^{1{\left(m-\gamma \right)}^{2}/2\varepsilon^{2}}. \end{array}$$

Each noise point of uniformly distributed noise appears randomly in the image, and the probability of occurrence is equal. Its probability density function is

(3) $$\begin{array}{c} \varepsilon =\frac{a+b}{2},\\ \gamma^{2}=\frac{{\left(b-a\right)}^{2}}{12}. \end{array}$$

In mathematical statistics, we generally do the difference between the estimated value of the parameter and the actual value of the parameter and then square the difference to take the mean of the square. This mean is called the mean square error and is denoted as MSE [15, 16]. In the field of image processing, the mean square error is often used, which can clearly show the changes of the image before and after processing:

(4) $$\begin{array}{c} \text{MSE}=\frac{1}{MN}\sum_{i=1}^{M}\sum_{j=1}^{N}{\left(k_{ij}-r_{ij}\right)}^{2}. \end{array}$$

Among them, *M* and *N* are the width and height of the image and *k*_*ij*_ and *r*_*ij*_ are the gray values of the points of the original medical image and the denoised medical image.

Peak signal-to-noise ratio (PSNR) is the most common and widely used objective measurement method for evaluating image quality, and its formula is

(5) $$\begin{array}{c} \text{PSNR}=10*\mathrm{lg}\left(\frac{255^{2}}{MSE}\right). \end{array}$$

The larger the value of PSNR, the smaller the difference between the images before and after processing. However, the PSNR value has no direct relationship with the subjective visual perception of the image.

Although we cannot calculate the total amount of information contained in an image, we can understand information entropy as the probability of certain information in the image. So, information entropy can be expressed by the following formula:

(6) $$\begin{array}{c} H=\sum_{i=0}^{255}p_{ij}\log\;p_{ij},\\ Pij=\frac{f\left(i,j\right)}{\left(M*N\right)}. \end{array}$$

Among them, *f*(*i*, *j*) is the frequency of occurrence of the gray value, and MN is the scale size of the image. Histogram equalization has an obvious effect on enhancing images with a small dynamic range. One of its biggest advantages is the ability to adaptively adjust the distribution of image gray levels, and its shortcomings are also obvious. The image is enhanced after histogram equalization processing. The effect is not easy to control, and it is possible to reduce the gray level of the image and make some details of the image disappear.

The article "Clinical and Imaging Study of Repetitive Transcranial Magnetic Stimulation in the Treatment of Morphine Dependence Through mGluR5/TDP43/NR2B Pathway" was retracted in 2022. Reason: concerns about the peer review.

To count the histogram in the original image, the formula is as follows:

(7) $$\begin{array}{c} p\left(r_{k}\right)=\frac{n_{k}}{n}. \end{array}$$

Calculate the cumulative distribution curve of the histogram; the gray scale transformation function is

(8) $$\begin{array}{c} S_{k}=\sum_{j=0}^{k}p_{r}\left(r_{j}\right)\\ =\sum_{j=0}^{k}\left(\frac{n_{j}}{n{}_{0}}\right). \end{array}$$

Use the cumulative distribution function to correct the original image, as shown in Figure 2.

For related medical images, the local contrast of pixels is positioned as

(9) $$\begin{array}{c} C_{ij}=\frac{\left|f_{ij}-\bar{f}\right|}{f_{ij}+f}, \end{array}$$

where $\bar{f}$ represents the average gray value of (*i*, *j*) 8 neighborhood pixels:

(10) $$\begin{array}{c} \bar{f}=\frac{1}{9}\sum_{k=i-1}^{k=i+1}\sum_{l=j-1}^{l=j+1}f_{kl}. \end{array}$$

The pixel gray value of the enhanced image is

(11) $$\begin{array}{c} f_{ij}=\left\{\begin{array}{cc} \bar{f}*\frac{1-C_{ij}}{1+C_{ij}}, & f_{ij}<\bar{f},\\ \bar{f}*\frac{1+C_{ij}}{1-C_{ij}}, & f_{ij}\geq \bar{f}. \end{array}\right. \end{array}$$

The image quality evaluated in this way will vary with the observer's experience and physical and psychological conditions. Therefore, subjective evaluation is generally not used as a stand-alone evaluation standard for image quality. It is also necessary to provide a more objective and objective evaluation method through objective evaluation methods. More intuitive data serve as an auxiliary reference, as shown in Table 1.

As an important method of measuring image quality, objective evaluation is to construct a quantitative index based on the human visual perception system and measure the image quality by calculating the size of the comparison index. Commonly used objective evaluation indicators include signal-to-noise ratio or peak signal-to-noise ratio, root mean square error, information entropy, and edge protection index.

## 3. Experiments and Results

### 3.1. Research Objects

We purchased 72 male healthy Wistar rats weighing 180–200g (7 weeks) from Beijing Weitong Lihua Experimental Animal Technology Co., Ltd. The breeding environment: room temperature of (22 ± 3 65289*e*, 12290). The breeding environment is quiet, the nursery cage is kept dry and clean, the rodent's activities are verified regularly every day, and any death or injury, with signs of disease, was removed in time.

Select the stimulus target: select the “8” RTMS head shape, and connect the center point of the two lines to the skull area near the excitatory motor cortex M1 of the cerebral hemisphere. Move the coil position and adjust. The tilt angle is used to find the best position to produce the maximum dynamic range of the engine (ME) at the bottom of the hybrid muscle. This is the goal of stimulation. Activation intensity of rTMS group: 80% exercise limit.

The article "Clinical and Imaging Study of Repetitive Transcranial Magnetic Stimulation in the Treatment of Morphine Dependence Through mGluR5/TDP43/NR2B Pathway" was retracted in 2022. Reason: concerns about the peer review.

Use TOYOBO Reverse Transcription Kit for cDNA synthesis. Configure the reverse transcription reaction solution according to the volume in Table 2. Add the total volume of the common reagents into one tube, and then evenly distribute it to each tube, on the icebox. Carry out the operation.

Detect the expression of NR2BmRNA by real-time fluorescent quantitative PCR, in a 0.2 ml PCR tube, and prepare the PCR amplification reaction system as shown in Table 3.

Carry out the RT-PCR reaction, repeat 3 times for each sample. After the reaction is over, store the sample at −20°C for later use. The reaction conditions are shown in Table 4.

### 3.2. Changes in Rats

The rats behaved more docilely during the morphine consumption period, were not irritable to stimulation, and had less aggressive behavior. After the morphine was removed, the rats showed grooming, sneezing, irritability, stiff tail, bowed head arched back, and hearing loss. The details are shown in Figure 3.

It can be seen that the withdrawal syndrome scores of the 2 h (10.42 ± 2.50), 6 h (15.42 ± 1.93), 12 h (9.25 ± 2.01), and 1 d (7.67 ± 1.92) groups of withdrawal syndrome were significantly higher than those of the normal control group (1.50 ± 0.80) (*P* < 0.05); the 6 h withdrawal group had the highest score and then gradually decreased. Three days after the drug was stopped, the behavioral indicators of rats decreased significantly, and some even disappeared. The score of withdrawal symptoms was similar to that of the normal control group, and the difference was not statistically significant (*P* > 0.05).

Under the microscope, it can be seen that NR2B protein has a large amount of expression in rat hippocampal neuron cells, the cell membrane shows circular fluorescent staining, and blue-stained cell nuclei can be seen in the fluorescent ring. A small amount of positive expression of NR2B protein can be seen in the normal control group, as shown in Figure 4.

The normal control group saw a small amount of positive NR2B protein-protein expression with a shade of fluorescence staining, with a significant increase in the mean fluorescence intensity of hippocampal NR2B in the 2 h, 6 h, 12 h, and 1 d withdrawal groups compared to the normal control group (378.56 ± 67.65); the difference had statistical importance (*P* < 0.05). The expression was also increased in the 3 d withdrawal group (437.24 ± 123.76); the difference was not statistically significant compared to the normal but there was no statistically significant difference in comparison with the control cohort (*P* > 0.05).

The article "Clinical and Imaging Study of Repetitive Transcranial Magnetic Stimulation in the Treatment of Morphine Dependence Through mGluR5/TDP43/NR2B Pathway" was retracted in 2022. Reason: concerns about the peer review.

We compared the brain changes under different loads of transcranial magnetic stimulation, as shown in Figure 5.

Compared with the baseline rest task, the main brain regions activated in the continuous attention task (before uncorrected) are the left supreme gyrus, right precuneus, left precuneus, right supreme gyrus, right middle occipital gyrus, left middle occipital gyrus, right middle temporal gyrus, right superior marginal gyrus, right talar fissure surrounding cortex, right auxiliary motor area, right dorsolateral superior frontal gyrus, right middle frontal gyrus, and left auxiliary sports area. Compared with the baseline rest task, the brain areas that are mainly activated for working memory tasks (before correction) are the right auxiliary motor area, left middle frontal gyrus, right orbital inferior frontal gyrus, right middle frontal gyrus, right hippocampus, and the lobules on the right side of the center, as shown in Figure 6.

### 3.3. Withdrawal Response and Protein Expression

Detox symptoms scores showed a positive correlation against NR2B hippocampal protein in expression levels (*r* = 0.522, *P* < 0.01), which suggested stable changes in NR2B in protein expression levels and detoxification syndrome in the postmorphine withdrawal, as illustrated in Figure 7.

We analyzed the correlation between the expression level of NR2B protein in the hippocampus of rats and the expression level of NR2BmRNA, as shown in Figure 8.

The results showed that the expression level of NR2B in the rat hippocampus was positively correlated with the expression level of NR2B mRNA (*r* = 0.746, *P* < 0.01), indicating that there was a constant change between the expression level of NR2B protein and the level of gene transfer.

## 4. Discussion

### 4.1. Behavioral Changes of Rats

The experimental results showed that there was no significant difference between the body weight of the rats in the morphine group and the normal control group. At the end of the experiment, it showed that the intake of low-concentration morphine solution had little effect on the food intake of rats, and it would not lead to insufficient fluid intake and nutrition. Therefore, we can analyze the difference in the detection indicators of rats in the morphine group, which is only caused by a factor such as morphine treatment, rather than brain damage caused by malnutrition and other diseases. Throughout the experiment, the morphine consumption of rats remained relatively stable, which further indicated that the changes in rat behavior and biological indicators after stopping the drug may be the result of repeated stimulation of the nervous system with morphine.

The article "Clinical and Imaging Study of Repetitive Transcranial Magnetic Stimulation in the Treatment of Morphine Dependence Through mGluR5/TDP43/NR2B Pathway" was retracted in 2022. Reason: concerns about the peer review.

This experiment also evaluated the withdrawal symptoms and severity of rats at 2 hours, 6 hours, 12 hours, and 1 day. Morphine was stopped after 3 days, which further verified the successful introduction of the morphine model. The results showed that the scores of withdrawal symptoms in the morphine group were 2 hours, 6 hours, and 12 hours, the morphine group was higher than the normal control group, and the difference was statistically significant. After 2 hours of morphine withdrawal, the incidence of the withdrawal syndrome in rats increased significantly, reaching the highest value of 6 hours of withdrawal and then beginning to decline. The first day of withdrawal was significantly higher than that of the normal control group. This result supports that rats suddenly withdraw after taking morphine for a long time, showing severe withdrawal syndrome.

### 4.2. Withdrawal Expression

The results show that long-term use of morphine can increase the expression levels of NR2B and NR2B mRNA protein. Significant increases were observed in the withdrawn group at 2 h, 6 h, 12 h, and 1 d compared to the normal control group, for which the differences were considered statistically significant. During the two-hour withdrawal period, there was a maximum content of this protein, and the number of expression levels decreased gradually with its duration. A statistically significant difference between the three-dimensional withdrawal with normal control compared to the three-dimensional segment was not observed. A large number of studies have shown that the use of morphine may cause the expression of NR2B to be regulated: the expression of NR2B in cultured rat C57 skin and hippocampal neurons increased significantly after 2 and 5 days of intermittent morphine treatment for several years after withdrawal; 2 weeks later, the expression level of NR2B protein increased significantly in the hippocampus of Wistar adult rats within 24 hours and 2 weeks after drug withdrawal and decreased to the reference level; and the results showed that the expression of NR2B and mRNA protein was significantly increased in the prefrontal lobe of rats after long-term morphine administration. The level of NR2B in the cortex and hippocampus increased. Regarding the expression of NR2B at the time of drug withdrawal, the results of different studies are inconsistent, which may be related to the way and time of administration of morphine.

The article "Clinical and Imaging Study of Repetitive Transcranial Magnetic Stimulation in the Treatment of Morphine Dependence Through mGluR5/TDP43/NR2B Pathway" was retracted in 2022. Reason: concerns about the peer review.

### 4.3. Repeated Transcranial Stimulation

With the analysis of functional magnetic collocation data, three types of comparisons are specifically to be included: comparison between a continuous work and a working basis, one between a working memory and a working basis, and one between a working memory and a continued work. Having only access to the patients' knowhow and then doing a *t*-test samples, the final continuance of attention working artifact activation maps and working memory decaying working artifact artifacts are largely reproduced in line with that of the previous ones. Therefore, the RVIP works selected in this study may be a good measure of sustained attention work and an auxiliary measurement of working memory tasks. High-frequency transboundary magnetic stimulation seems to mainly reduce the signal in these areas of the brain. It mainly includes the following areas of the brain: upper left ring, left atrium, right atrium, right middle frontal ring, and left cerebellum. The cerebral cortex has always been a necessary part of continuous attention.

## 5. Conclusion

Repetitive transcranial stimulation is to use the magnetic field generated by the transient current in the excitation coil to excite the induced current in the coil, determine the target area of the patient's brain, and adjust the stimulation parameters, such as intensity, pulse frequency, and pulse number to control the cortex to stimulate the target area. The pathological changes caused by the long-term use of morphine are most obvious in brain injury. In the early stage of the experiment, after the rats were dependent on morphine, the related changes of NR2B hippocampal expression and epigenetic modifications and hypotheses related to morphine withdrawal syndrome changed. The change in the acetylation level of H3K9 cells in the promoter region of the gene may be one of the mechanisms of morphine withdrawal syndrome. Based on previous studies, the genetic modification of the NR2B stick is further studied, and the reward pathway is involved. Other areas of the brain, such as the nucleus and abdomen, will also provide more information through research to understand the relevant mechanisms of morphine dependence. The authors of this paper lack many aspects because the sample number and are not very large. It will cause the instability of behavioral effect and image effect. Second, the drug phenomenon of cross-border magnetic stimulation has not been well dealt with. In order to eliminate the influence of cross-border magnetic stimulation simulation drugs, this study sets up a control group. However, the research center does not have a special pseudo-stimulation coil. This kind of fake stimulation coil can generally achieve a very realistic effect. When it stimulates the subject's brain, the subject will have a certain sense of vibration.

The article "Clinical and Imaging Study of Repetitive Transcranial Magnetic Stimulation in the Treatment of Morphine Dependence Through mGluR5/TDP43/NR2B Pathway" was retracted in 2022. Reason: concerns about the peer review.

## Figures and Tables

**Figure 1:** EEG International Electrode location.

**Figure 2:** Original image correction. (a) Histogram equalization. (b) Linear transformation. (c) Piecewise linear transformation.

**Figure 3:** Different withdrawal time scores.

**Figure 4:** Changes in different withdrawal times.

**Figure 5:** Different loads stimulate intracranial changes.

**Figure 6:** Comparative activation of working memory task and continuous attention task.

**Figure 7:** NR2B protein expression level.

**Figure 8:** NR2B protein expression level and NR2BmRNA expression level.

**Table 1:** Data auxiliary table.

Level	Relative scale	Absolute scale
1	Relatively best to be evaluated	Well
2	Better than the average to be evaluated	Slightly better
3	Average level to be evaluated	General
4	Worse than the average to be evaluated	Slightly worse
5	Relatively worst to be evaluated	Very bad

**Table 2:** Reverse transcription reaction system.

Composition	Volume (*µ*l)	Final concentration
DNAse treated RNA	4	—
5 × buffer	4	1
dNTPs (10 mM)	1	0.5 mM
Oligo (dT)18 (50 *μ*M)	1	25 pM
Random primer (100 *μ*M)	0.5	25 pM
MMLV reverse transcriptase (200 U/*μ*l)	1	10 U/*µ*l
DEPC H2O	8.5	—
Total volume	20	—

**Table 3:** PCR amplification reaction system.

Composition	Volume (*µ*l)	Final concentration
cDNA	1	—
Primer *f* (10 *µ*M)	0.5	20 pmol/*µ*l
Primer *r* (10 *µ*M)	0.5	20 pmol/*µ*l
2 × mix	12.5	1×
SYBR Green I (10×)	1	0.4×
ddH2O	9.5	—
Total volume	2.5	—

**Table 4:** Reaction conditions.

NR2B				GAPDH		
Experimental steps	Temperature	Time	Number of cycles	Temperature	Time	Number of cycles
Predenaturation	94°C	2 min	35	94°C	2 min	35
Transsexual	94°C	30 sec		94°C	30 sec	
Annealing	52°C	30 sec		55°C	30 sec	
Extend	72°C	30 sec		72°C	30 sec	
Extend	72°C	10 min		72°C	10 min	

## Data Availability

The data that support the findings of this study are available from the corresponding author upon reasonable request.
